# Systematic Review on Multilevel Analysis of Radiation Effects on Bone Microarchitecture

**DOI:** 10.1155/2022/9890633

**Published:** 2022-06-06

**Authors:** Ayuni Amalina Abu Bakar, Noor Shafini Mohamad, Mohd Hafizi Mahmud, Hairil Rashmizal Abdul Razak, Ann Erynna Lema Thomas Sudin, Solehuddin Shuib

**Affiliations:** ^1^Centre of Medical Imaging, Faculty of Health Sciences, Universiti Teknologi MARA Selangor, 42300 Bandar Puncak Alam, Selangor, Malaysia; ^2^Medical Imaging Program, College of Medicine and Health, St Luke's Campus, University of Exeter, EX1 2LU Devon, UK; ^3^Faculty of Mechanical Engineering Universiti Teknologi MARA Shah Alam, 40450 Shah Alam, Selangor, Malaysia

## Abstract

**Introduction:**

Modern radiation therapy has become an effective method to treat and monitor tumour growth in cancer patients. It has proved to be a successful way to minimise mortality rates. However, the adverse effects of radiation have been historical evidence in the clinical environment involving diminishing the quality and density of bone and causing fragility fracture to the bone in the long run. This systematic review was aimed at identifying and evaluating the effects of irradiation on morphology and mechanical properties of murine model bone in previous publications.

**Methods:**

A systematic literature review was undertaken following the Preferred Reporting Items for Systemic Reviews and Meta-analysis (PRISMA) guidelines. A comprehensive literature search was performed using Scopus, Web of Science, and Science Direct databases (English only studies published between 2015 and 2020). The selected studies were evaluated according to three criteria: (1) criteria for study sample selection; (2) criteria for methodological procedures; and (3) criteria for detection and evaluation.

**Results:**

The initial search strategy identified 1408 related studies, 8 of were included based on inclusion and exclusion criteria. This review revealed an association between bone destruction and the magnitude of time and dose postirradiation. We agreed that the effect of radiation on bone morphology and strength primarily is a later stage event but noticeable in both low (1 Gy) and high dose (30 Gy) radiation. Trabecular and cortical bone microstructures were significantly altered at irradiation and contralateral sites. Besides, the mechanical strength was significantly impacted in both shorter and longer periods.

**Conclusion:**

Overall, the radiotherapy altered bone microstructures and substantially decreases bone mechanical properties. The alteration was related to quantity and the activity of the osteoblast and osteoclast. Early detection of those most at risk for radiation-induced bone alterations could lead to better prophylactic intervention decisions.

## 1. Introduction

Current ionising radiation therapy regimen is considered as an effective method for treating cancer. Cancer patients have been given low dose exposure from radiation therapy to ensure sufficient tumour control [1]. Approximately, 2/3 of cancer patients received radiation therapy associated with other treatment such as surgery [1]. This treatment has proved to be a successful way to minimise mortality rates and reduce pain from the bone metastases.

However, radiation therapy was reported to have adverse effect of diminishing the quality and density of bone, causing fragility and fracture to the bone in the long run [2–4]. More than 65% of women treated for various pelvic tumours have hip fracture five years postradiotherapy. Tennenbaum et al. [5] stated that 20% of normal osteoporosis patient with fragility fracture reported mortality due to long term hospitalisation. Fixation implant treatment would be impossible on the osteoporosis patient due to weak bone structure.

Although the effect of posttherapy causing bone degradation of bone architecture is known [6], skeletal changes in irradiated osteoporosis femur related to morphological, mechanical, and tissue properties have not generally been explored in ex vivo animal model. This literature review provides a thorough overview on the effect of irradiation on morphological, mechanical, and tissue properties of ex vivo murine model.

The current review, therefore, was aimed at providing knowledge and promoting better understanding of ionising radiation's impact on multilevel bone mechanical and tissue properties of murine model bone.

## 2. Methodology

We followed the protocol of Preferred Reporting Items for Systematic Reviews and Meta-analyses (PRISMA), i.e., formulation of research questions, systematic review process for selecting the articles (identification, screening, and eligibility), quality appraisal, data abstraction, and analysis.

PRISMA is usually used in medical research; the inclusion and exclusion criteria for a specific study may be identified simultaneously [7]. PRISMA is useful as standard healthcare guidelines [8]. PRISMA also highlights the review report, which analyzes randomised trials that are also important for reporting systematic reviews for other studies [9].

### 2.1. The Databases

The databases chosen were Scopus, Web of Science (WoS), and Science Direct because these databases are robust and cover more than 256 fields of studies, including health sciences. Precisely, in Scopus indexes, a total of 65 journals are related to radiology. In addition, they are trustworthy databases. However, to increase the possibility of finding relevant papers, it is recommended that authors perform their selection process using more databases [10].

### 2.2. Formulation of Research Question

The research question formulation was based on PICo tool, which are population or problem, interest, and context. We have included ex vivo murine model (as the population), the effect of irradiation (interest), and morphological, mechanical, and tissue properties (context), which then formulate into the main research question: to investigate the effect of irradiation on morphological, mechanical, and tissue properties of bone using an ex vivo murine model.

### 2.3. The Systematic Review Process for Selecting the Articles

The systematic review process for selecting the articles consists of identification, screening, and eligibility stages. The flow chart of study selection process is presented in Figure 1.

#### 2.3.1. Identification

The first stage is identifying keywords, followed by searching on thesaurus, dictionaries, encyclopaedia, and past analysis for related and similar meanings. Both US and UK terms were used, such as “ionizing” and “ionising.” The full search string for each database is recorded in Table 1.

#### 2.3.2. Screening

The identified papers' titles, abstracts, keywords, authors' names, and year of publication were exported to an Excel spreadsheet during the screening stage. Two reviewers independently assessed the titles and abstracts of the selected articles based on several inclusion and exclusion criteria (Table 2). Five years' timeline from 2015 to 2020 was selected for the timeline. Related articles with full texts were downloaded and brought to eligibility stage.

#### 2.3.3. Eligibility

The two researchers then independently evaluated eligibility by carefully scanning the entire articles. The titles, abstracts, and keywords of all the articles were reviewed to ensure that they met the inclusion criteria. Disagreements between the researchers were discussed and resolved during this process. If no agreement could be made, a third reviewer's opinion was sought. Lastly, an experimental study using a murine model to quantify the changes in bone properties was included. The experimental methodology must include bone microarchitecture assessment using micro-CT scanning.

### 2.4. Quality Appraisal

The quality appraisal is an assessment of methodological quality. It allows evaluating quality and susceptibility, which is essential when interpreting research or conducting systematic reviews [12]. For the articles to be included, it is recommended that researchers classify the remaining articles into three qualities: high, moderate, and low [13]. Only articles classified as high and moderate are to be reviewed.

In this review, the critical appraisal process was carried out using a randomised controlled trial structured checklist by Quality Appraisal Skill Programme (CASP) (adapted from Guyatt et al. [14]). Eleven questions assist authors in rating the quality of articles systematically. The first three questions were screening questions that can be answered quickly. If the answer to all questions is “yes,” the remaining questions are worth continuing.

Finally, the remaining papers were submitted to the two researchers for quality evaluation to ensure the articles' quality content. Both researchers must mutually agree that the quality must be at least at a moderate level. Any disagreement was discussed between them before deciding on the inclusion or exclusion of the articles for the review.

## 3. Results

### 3.1. Background of the Selected Articles

From the three databases, 1408 articles were retrieved in the first stage of the systematic review process. All articles were screened based on inclusion and exclusion criteria; duplicate articles were also eliminated. Overall, a total of 1025 articles were excluded, and a balance of 375 articles was assessed for eligibility. The titles, abstracts, and keywords of the articles were extensively reviewed to ensure that they met the inclusion criteria and were appropriate to be included in the current study. 367 articles were removed because the empirical evidence was not focused on the radiation effect on mice bone morphology and mechanical properties. Finally, a total of eight remaining articles are available for evaluation (Table 3). The methodology applied was listed in Table 4.

### 3.2. Main Findings from Reviewed Articles

This study was focusing only on the bone microstructures, strength, and tissue properties. Bone histomorphometry was excluded from this research since it is out of the research question.

The study by Bartlow et al. [16] provided data that radiotherapy reduces bone morphology and bone fracture durability. In general, relative alterations in the morphology of mid-diaphysis cortical bone after irradiation were less severe compared to changes in bone fracture strength. Mice were exposed to the radiation *in vivo* and ex vivo using devitalised tissue of mice strain (BALB/cJ). During *in vivo* irradiation, the mice received fractionated irradiation (4 × 5 Gy) while *ex vivo* femur was subjected to a single dose of 20 Gy. Fractionated dosing for devitalised bone was unnecessary because there were no living cells capable of repairing the DNA damage. The control mice group was compared with 0-, 4-, 8-, and 12-week postirradiation group (*n* = 15/group/time point).

Overall, *μ*CT scanning results showed relative alteration in mid-diaphyseal cortical bone morphology in 8 and 12 weeks but not in the early week. At 4-, 8-, and 12-week postirradiation, there was a reduction in cortical thickness. In comparison, irradiation at any time period did not significantly impact the total area (Dp Tt.Ar). Compared to the control group, the endosteal area increased at 4-, 8-, and 12-week postirradiation. Similarly, fracture toughness changes—determined using devitalised mice cadaver femurs—found that cortical bone toughness was reduced in the early weeks after the radiation, but no further reduction occurs after. Irradiation of devitalised femurs also decreased fracture toughness (-29%) to a lesser degree than that seen *in vivo*. This is because fracture toughness improved over time due to the bone recovery.

Wright et al. [17] conducted a study to explore radiation-induced bone loss in local and systemic effects on bone. They examined the impact of irradiation on bone volume and microarchitecture using *μ*CT. The right hindlimb represents the irradiation sides compared to the left hindlimb (contralateral-shielded bone) and control bone. A single dose of 2 Gy was administered using an X-ray machine. One-week postirradiation, BV/TV in irradiated hindlimbs was decreased by 22% in the tibia and 14% in the femur compared to the control group. These alterations in irradiated bone were significant compared to changes found on the contralateral side. The BV/TV of contralateral tibiae in irradiated hindlimb was decreased by 17% compared to control. Besides, there was a reduction in Conn. D (-50%) and Tb.N (-16%) and 20% increase in Tb.Sp of the irradiated hindlimb compared with the control group. The same patterns were found at the contralateral bone sites. Nevertheless, the cortical bone properties did not change significantly between the groups.

Another relevant study by Limirio et al. [15] investigates the ionising radiation's effect on bone morphology and bone strength on Wistar rats. The rats were divided into four groups depending on the euthanisation period (*n* = 5): control 30 days (C30), irradiated 30 days (IR30), control 60 days (C60), and irradiated 60 days (IR60). Single 30 Gy of radiation was administered to the left leg. The right legs were not radiated and assigned as the control group. 30 Gy was chosen since it is believed to cause bone damage, so the effect of radiation on the bone can be studied [21, 22]. They found that radiation impaired bone quality and reduced strength. In addition, the findings indicated that the harmful consequences of radiation increased in later time periods. Data from *μ*CT demonstrated that C60 had the highest radiodensity than other groups because bone became denser than in earlier times. The radiodensity of IR30 and IR60 reduced by 9% and 20%, respectively (Figure 2). Biomechanic analyses showed degeneration, damaged bone wholeness, and reduced resistance to fragility fractures. Flexural and elastic modulus values have been reduced in the radiated groups relative to the control groups. However, there were no changes in flexural strength between the control and radiated groups.

A study by Barbosa et al. [18] investigated 30 Gy radiotherapy's effects on biomechanical, histomorphometric, and microstructural features of rabbits. Adult male New Zealand rabbits (*n* = 18) were randomly assigned into six groups: a control group and five irradiation groups euthanised after 24 hours (Ir24h), 7 days (Ir7d), 14 days (Ir14d), 21 days (Ir21d), and 28 days (Ir28d). The researchers found that ionising radiation changes the microarchitecture of cortical bone and increases bone fragility compared to the control bone. There are slight reduction of the Ct.Th, Ct.V, and Ct.Po from day 7 to day 28 postirradiation (Figure 3). However, these changes were only significant at the later period (14 and 21 days) and not instantly after the exposure to the radiation. The biomechanical test results demonstrated reduced force, work to failure, and stiffness in the irradiation group compared to the control group. However, a significant difference compared to the control group was evidenced for rabbits sacrificed after 14 days for force and 21 days for work for failure and stiffness. Besides, rabbits euthanised after 21 and 28 days have significantly lower parameters studied than rabbits euthanised after 24 hours.

Additionally, results from *μ*CT demonstrated bone alteration on the more extended period postirradiation. The significant difference in Ct.V is only shown 21 days postirradiation. Furthermore, there is a significant Ct.Th reduction on the 21 and 28 days compared to 24 hours postirradiation. Apart from that, the Ct.Po values observed 28 days postirradiation were significantly higher than values obtained from animals sacrificed after 24 hours. Taken together, they conclude that the effect of radiation is more noticeable in the later period.

Study regarding the early and delayed effect of a single low dose of total-body exposure on bone microarchitecture was done by Barbosa et al. [18]. To explore this phenomenon, 16 weeks of BALB/c mice were randomly divided into four groups depending on the exposure dose (0.17 Gy, 0.5 Gy, 1 Gy, and 0 Gy represent the control group). Then, mice from each group were divided into two euthanised periods: three days (early effect) and 21 days (delayed effect) postirradiations. The significant changes to bone microarchitecture were only evident when the mice are exposed to 1 Gy dose. On the contrary, there was no cortical bone geometry alteration when the mice were exposed to low dose effect (0.17 Gy and 0.5 Gy) at day 3 or 21 postirradiation. Histogram of the radiation effects on trabecular bone was displayed in Figure 4. The 1 Gy group shows a significant reduction in BV/TV by 21% and Conn.D by –22% on day 21 compared to the control group, whereas Tb.Sp increased by 9%. Besides, on day 21, Conn.D was significantly reduced by 21% when mice are being exposed to 0.17 and 1 Gy radiation.

Likewise, Oest et al. [19] investigated the early and later effect of radiation in bone microarchitecture locally and contralaterally. 160 BALB/cJ mice (*n* = 10/group) were administered with 4 × 5 Gy of radiation and divided into the euthanisation period: 0, 1, 2, 4-, 8-, 12-, and 26-week postirradiation. They found that reducing BV/TV in the irradiated femurs was evident after 4-week postirradiation and not in the earlier week. Notably, there was a reduction in BV/TV and Conn.D for both the irradiation and control groups. However, the reduction was more significant and rapid in the irradiation group compared to the control group. Precisely, there was an increase in BV/TV in the early week (0, 4 days) followed by a rapid reduction of BV/TV for the irradiation group later. The contralateral group also followed a similar reduction pattern. In contrast, Ct.Ar kept increasing over time for all groups. However, for irradiation and the contralateral groups, the increase rate was lesser relative to the control group. The mechanical strength test result showed that irradiation groups have less strength and stiffness than the control group. The reduction in bending strength for the irradiation group occurred in 2 to 8 weeks postirradiation. Precisely, at 12 weeks, there were reductions in 14.1% of bending strength, 13.3% in stiffness, and 13.5% bending strength of the irradiation group compared to the control group. It appeared that at this specific time, the bone might have a greater risk of fracture.

Sullivan et al. [20] revealed a reduction in BV/TV (-41%), Tb.Th (-24%), Tb.N (-35%), and cortical stiffness (-32%) in the irradiated ovariectomy mice compared to the sham group on the 35 days postirradiation. Conversely, Ct.Th follows the opposite pattern as in the irradiated group shown increased by 33% compared to the sham group. Additionally, nonovariectomy also follows the similar reduction pattern in the BV/TV (-46%), Tb.Th (-10%), Tb.N (-30%), and cortical stiffness (-29%) compared to the control group. The researchers administered a fractionated dose of 3 × 6 Gy to 13-week C57BL mice. The trabecular bone in the OVX+IRR seems more porous and lower in quantity compared to another groups (Figure 5).

In addition, study from Zhai et al. [22] revealed the effect of radiation on both a single 2 Gy dose and consecutive 3 × 8 Gy. Mice were euthanised on days 3, 7, 14, 30, and 60 postirradiation to study the immediate and latent effects of the radiation. As early as 7 days after radiation, the single 2 Gy local irradiation model mice demonstrated impaired trabecular and cortical structure in the locally irradiated and contralateral femur (Figure 6). The femoral bone was fragile, with a huge decline in BV/TV, Tb.Th, Tb.N, and Ct.Th, as well as a significant rise in Tb.Pf. Precisely, there was a reduction in BV/TV in the directly irradiated femur (-35%) and contralateral femur (-17.82%) compared to the control femur. Besides, they revealed a reduction in Ct.Th in the directly irradiated femur (-9.03%) and contralateral femur (-4.33%) compared to the control femur. In contrast, Tb.Sp in trabecular bone was substantially elevated in the directly exposed femur (+21.96%) and contralateral femur (+18.94%), respectively.

Nevertheless, the alterations in bone morphometrics had restored substantially at 30 days postirradiation at both local and contralateral femur. Similarly, there was destructed in direct and contralateral trabecular bone in 3 × 8 Gy on day seven postirradiation. The directly irradiated mice had lower BMD, BV/TV, and Tb.N, while the contralateral femur had lower BMD but higher Tb.Sp. Moreover, bone loss and architectural destruction in the directly irradiated femoral bone remained 60 days after irradiation.

## 4. Discussion

### 4.1. Overview

Modern radiation therapy has become an effective method to treat and monitor tumour growth in bone metastases patients. Radiation therapy has proved to be a successful way to minimise mortality rates [17]. However, the degenerative effects of radiation in the clinical environment have been historically evident. Aside from its remarkable ability to treat and cure cancer, radiation therapy is also known to destroy cells and impairs their function [23]. The adverse effect involves diminishing the quality and density of bone, causing fragility and fracture to the bone in the long run. In addition, large radiation doses used to treat cancer have been strongly linked to osteoradionecrosis [24]. In most of the reviewed studies, *μ*CT and FE analyses were used to quantify the bone properties. *μ*CT is most commonly used in previous literature [15–22] since it is considered as a gold standard for the assessment of preclinical animal studies [25].

### 4.2. Immediate and Latent Radiation Effect

The research articles that have been reviewed clearly show that radiation causes bone destruction depending on time and dose. The effect of radiation on bone morphology and strength was more noticeable at a later stage [15, 16, 18, 21]. The studies have consistent results with one another. Bartlow et al. [16] showed changes in Ct.Th and endosteal area only at 4, 8, and 12 weeks postirradiation but not in 0 week. A study on the low dose from Lima et al. [21] showed no alterations in cortical and femur trabecular bone morphology at day 3, but changes were only observed on day 21. Likewise, Limirio et al. [15] found that reduction of the radiodensity is more prominent in the later period, which is on day 60 than day 30. Barbosa et al. [18] complemented the previous finding since they demonstrated that IR changes the microarchitecture of cortical bone and increases bone fragility compared to the control bone. However, these changes were seen only at the later period (e.g., 14 and 21 days) and not instantly after the exposure to the radiation (1- and 7-day postirradiation).

Nonetheless, the study from Zhai et al. [22] is in contrast with the previously discussed study. They revealed that destruction on trabecular and cortical bone local and contralateral femur was evidence in both early (7 days) and latent time (60 days) postirradiation. The alteration was initially evidenced as the breakdown of trabecular bone and the reduction of bone quantity continue over a long period after radiation exposure. Furthermore, the trabecular bone was clearly fragile and brittle in both single and 3 consecutive 8 Gy of radiation.

### 4.3. Low and High Dose Radiation Capable in Inducing Bone Loss

We found that the radiation effects on bone morphology and strength were evidenced in both low and high radiation. Wright et al. [17] showed the trabecular bone parameter alteration when the bone was exposed to low radiation of 2 Gy as early as a week postirradiation. However, there was no alteration in cortical bone detected. Besides, bone deterioration has been documented at irradiation sites and contralateral sites, proving that both local and systemic impact of irradiation has harmful effects on the bone. These results are in compliance with the clinical records of a systemic osteopenia cancer patient that received radiotherapy [26, 27]. The complication of radiation at the distant bone and nonskeletal locations might be due to vascular damage and inflammation [26, 27]. Lima et al. [21] reported similar results previously recorded by Wright et al. [17] and Bartlow et al. [16]. According Lima et al.'s [21] study, a very low dose of 1 Gy radiation can cause significant changes to bone microarchitecture on day 21 postradiation. They conclude that low-dose radiation can damage mesenchymal stromal cells as early as day 3 after exposure, which may explain the radiation's later destructive effects on bone quality. Besides, the osteoclast number increased on day 3 of postradiation. Willey et al. [28] showed similar results, which show osteoclasts and changes in bone resorption activity after irradiation within three days after 2 Gy of radiation. This result is consistent with the histomorphometry finding from a study done by Oest et al. [19].

Likewise, the study from Zhai et al. [22] revealed that single 2 Gy dose and three consecutive 8 Gy dose cause a prolonged decline in bone quantity and destruction in bone microarchitecture. However, the bone deterioration induced by a single 2 Gy dose of local radiation is likely to regenerate entirely, but the bone impairment induced by three 8 Gy doses of local radiation occurs faster, lasts longer, and is difficult to recover.

Additionally, previous *in vivo* studies found that ionising radiation at dose 30 Gy severely altered the microarchitecture in osteoporosis bone [15, 18, 28–30]. The bone is more porous, increasing the bone's space, which is inevitable in mice bone. Several previously reported studies showed the harmful impacts of radiation on the bone [32], while some have demonstrated positive effects on osteoblastic differentiation and bone-specific gene expression [33]. In addition, Ma and Shen [23] reported radiation damages bone quality and quantity by reducing cell functions and blood circulation. Similarly, Green et al. [34] reveal that radiation alters the balance between bone resorption by osteoclasts and bone creation by osteoblasts, resulting in lower mineralization.

### 4.4. Radiation-Induced Bone Loss: Bone Cell Activity (Osteoblast and Osteoclast)

The theory for mechanism in alteration of bone postradiation is circling around the destruction of small blood vessels, inducing hypoxia and disrupting osteoblast and osteoclast activity. Normal bones required a consistent blood supply for nutrients and support. Blood supply damage presents in three stages in bone tissue following radiation: hypoxia, hypocellularity, and hypovascularity [36]. Eventually, the amount of functioning structural elements that work will be reduced causing bone atrophy. Moreover, osteoclast progenitors in the bone marrow are radiosensitive due to the high proliferative rate, and their deficiency may cause osteoclast loss in the long run [38]. The osteoclast is important in maintaining the bone remodelling process. Macrophage and neutrophil will be activated when there is any injury or death of cells in the bone marrow. Since osteoclasts are associated with macrophages, they are also triggered to promote rapid bone loss.

Besides that, it is reasonable to hypothesise that radiation causes impairment in bone through alteration of mesenchymal stromal cell fate. Wright et al. [17] revealed that the amount of osteoclast increased one week postirradiation might be one of the possible factors in reducing bone volume. In addition, Oest et al. [19] showed an early elevation in osteoclast quantity at one to two weeks postradiation, followed by a long osteoclast reduction [37]. Lima et al. [21] confirmed that radiation exposure inhibited stromal cell development into osteoblasts on day three postradiation. They suggest that radiation may damage bone growth by impairing the proliferation and differentiation of osteoclast progenitors. Consistent with these reports, Willey et al. [28, 38] found that osteoclast activation occurs three days after irradiation, and most bone destruction occurs 7–10 days afterwards. They detect significant elevation in osteoclastogenesis only three days after entire body exposure. Once trabecular connections are destroyed, they can no longer transmit the mechanical loads required for bone repair communication. Likewise, the study by Oest et al. [39] found an increased osteoclast number as early as one week prior to the irradiation. They believed that higher osteoclast counts corresponded with higher trabecular resorption.

### 4.5. Radiation-Induced Bone Loss: Growth Plate Activity

Little is known about the role of growth plate activity in radiation-induced bone loss. This might be one possible explanation regarding the alteration in bone microstructures. A previous study of the radiation effect on tibia growth plate showed disruption of wide regions of the growth plate with chondrocyte areas and a drastically decreased calcification zone postirradiation [32]. Growth plate chondrocytes have a high mitotic index, making them vulnerable to radiation-induced tissue damage [42]. Moreover, injury to the bloodstream in the metaphysis and chondrogenesis arrest in the growth plate may have caused changes in the calcification zone.

### 4.6. Local and Systemic Effect of Ionising Radiation

There is evidence of a local and systemic impact on trabecular bone destruction after radiation, with bone loss deterioration occurring in the irradiated and contralateral nonirradiated regions. Thus, the process of systematic bone loss following local irradiation must be explored to establish cancer patient prevention and therapy techniques. A study by Zhai et al. [22] revealed that rapid bone loss destruction and reduction of bone quantity could manifest as both local and systemic impacts at three days postradiation for low 2 Gy doses and three 8 Gy doses. Additionally, microCT demonstrated that the irradiated femur and the contralateral femur had considerably thinner compact bones than the control group. Precisely, there was a reduction in BV/TV in the directly irradiated femur (-35%) and contralateral femur (-17.82%) compared to the control femur. By contrast, Tb.Sp in trabecular bone was substantially elevated in the directly exposed femur (+21.96%) and contralateral femur (+18.94%), respectively.

A study from Zhang et al. [41] provided new perspectives for the underlying mechanisms of local and systemic bone loss. Bone loss caused by ionising radiation is associated with increased bone resorption, triggered by a raised iron content in the body and direct activation of osteoclast development. Iron metabolism and bone homeostasis are strongly connected. Iron overload promotes osteoporosis with enhanced osteoclastogenesis, demonstrated by increased bone resorption and decreased bone production [42]. In healthy postmenopausal women and middle-aged men, increased iron storage level is linked to increased bone loss [43]. These findings imply that increased iron levels may be a risk factor for rapid bone loss. Taken together, recent research shows that total body irradiation raises serum iron levels in mice and can last for three weeks or more [41, 44].

### 4.7. Strengths and Weaknesses of This Review

This systematic review focused on the radiation effect on bone microstructures and strength using *μ*CT, FEA, and 3-point bending test. Other aspects such as histomorphometry analysis and bone marrow stromal cell cultures were not being explored. Histological analyses are recommended in the future study since it may be helpful to understand the impact of cellular activity (osteoclasts and osteoblasts), extracellular matrix changes (alignment and cross-linking), and radiation-induced bone loss. Histomorphometry studies allow us to correlate cell structure to their specific function.

Strengths of the studies included using *μ*CT, which is considered as a gold standard for the assessment of preclinical animal studies [25]. It is most commonly used in previous literature [15–19]. Mechanical testing such as FEA and 3-point bending tests was frequently used to study bone integrity.

## 5. Conclusion

Radiation causes bone destruction early and latent time. It is expected that the current standards of care of radiation therapy could significantly improve by targeting the bone microenvironment to treat cancer patient. Many preclinical studies have shown that an increase of the osteoclastic bone resorption will contribute to the development of bone cancer [45–47]. Significantly, early alteration of cortical and trabecular bone microstructures can be related to the quantity and the activity of the osteoblast and osteoclast. Early detection of those most at risk for radiation-induced bone alterations could lead to better prophylactic intervention decisions.

## Figures and Tables

**Figure 1:** Flow chart of study selection process (adapted from Shaffril [11].

**Figure 2:** Radiodensity analysis results. Image courtesy from Limirio et al. [15].

**Figure 3:** The mean and SD value of morphologic parameters measured by *μ*CT for Nir and IR bone sacrificed after different time. (a) Ct.Th, (b) Ct.V, and (c) Ct.Po. Image courtesy from Barbosa et al., [18].

**Figure 4:** Radiation effects on trabecular bone microarchitecture at days 3 and days 21 as measured by *μ*CT. Image courtesy from Lima et al. [21].

**Figure 5:** 3D image representation of the trabecular bone (pink) and cortical bone (grey). (a) NONOVX+NR, (b) NONOVX+IRR, (c) OVX+NR, and (d) OVX+IRR. Image courtesy from Sullivan et al. [20].

**Figure 6:** 3D image representation of the femur at 7 and 30 days post single 2 Gy direct irradiation. (a) 7 days and (b) 30 days postirradiation. (A) Coronal cross-sectional femur, (B) 3D femoral trabecular bone, and (C) 3D femoral cortical bone. Image courtesy from Zhai et al. [22].

**Table 1:** Database search string.

Database	Search string
WoS	(((TS = (ioni?ing radiation effect∗)) OR TS = (microarchitecture properties micro strength mechanical micro computed tomography)) AND TS = (mice mouse bone)) NOT TS = (spacelight space)
Scopus	TITLE-ABS-KEY ((“RADIATION EFFECT∗” OR “RADIATION IMPACT” OR “IONISING RADIATION” OR “GAMMA RADIATION “OR irradiation) AND (gamma OR ionizing) AND (mouse OR mice) AND (mechanical OR strength OR “MICRO CT” OR “MICRO COMPUTED TOMOGRAPHY”) AND (bone))
Science Direct	Radiation Effect Ionising Radiation Mice Mouse Bone Strength Mechanical Micro

**Table 2:** The inclusion and exclusion criteria.

Criteria	Inclusion	Exclusion
Literature type	Journal (research articles)	Journals (review), book series, book, chapter in book, conference proceeding
Language	English	Non-English
Timeline	From 2015 to 2020	<2015
Subject area	Health science, mechanical engineering	Other than health science, mechanical engineering
Keywords	Radiation, irradiation, effect, Ionising, mice, mouse, bone, strength, mechanical, micro, gamma, micro computed tomography	Space, spacelight

**Table 3:** Reviewed studies that have been selected.

Author, years	Titles
Limirio et al., [15]	Ionising radiation and bone quality: time dependent effects
Bartlow et al., [16]	Limited field radiation therapy results in decreased bone fracture toughness in a murine model
Wright et al., [17]	Single-limb irradiation induces local and systemic bone loss in a murine model
Barbosa et al., [18]	Effect of ionising radiation after-therapy interval on bone: histomorphometry and biomechanical characteristics
Oest et al., [19]	Longitudinal effects of single hindlimb radiation therapy on bone strength and morphology at local and contralateral sites
Sullivan et al., [20]	A mouse model for skeletal structure and function changes caused by radiation therapy and oestrogen deficiency
Lima et al., [21]	Exposure to low-dose X-ray radiation alters bone progenitor cells and bone microarchitecture
Zhai et al., [22]	Influence of radiation exposure pattern on the bone injury and osteoclastogenesis in a rat model

**Table 4:** Methodology of reviewed studies.

Citation	Rodents' strain and sample size (*n*)	Radiation dose	Modalities used	Timing of data collection post irradiation
Limirio et al., [15]	Wistar rats *n* = 5	30 Gy	(1) *μ*CT (2) Mechanical testing	Day 30 and 60
Bartlow et al., [16]	BALB/cJ *n* = 15	20 Gy	(1) *μ*CT (2) Fracture toughness testing	Weeks 0, 4, 8, and 12
Wright et al., [17]	C57Bl/6 *n* = not described	2 Gy	*μ*CT	Day 7
Barbosa et al., [18]	NZ rabbits *n* = 6	30 Gy	(1) *μ*CT (2) Mechanical testing	Day 1, 7, 14, 21, and 28
Oest et al., [19]	BALB/cJ *n* = 10	4 × 5 Gy	(1) *μ*CT (2) Mechanical testing	Weeks 0, 1, 2, 4, 8, 12, and 26
Sullivan et al., [20]	C57BL/6 *n* = 8	3 × 6 Gy	(1) *μ*CT (2) Mechanical testing	Day 35
Lima et al., [21]	BALB/cBYJ *n* = 17 and 18	0.17 Gy, 0.5 Gy, and 1 Gy	*μ*CT	Day 3 or 21
Zhai et al., [22]	Male Sprague-Dawley rats *n* = 6	2 Gy and 3 × 8 Gy	*μ*CT	3, 7, 14, 30, and 60 days

## Data Availability

The data supporting this systematic review are from previously reported studies and datasets, which have been cited.
